# Prominin 1 Significantly Correlated with Bone Metastasis of Breast Cancer and Influenced the Patient's Prognosis

**DOI:** 10.1155/2022/4123622

**Published:** 2022-06-25

**Authors:** Cheng-cheng Yu, Yi-nan Wu, Kai-min Hu, Su-zhan Zhang

**Affiliations:** ^1^Department of Orthopedic Surgery, The Second Affiliated Hospital, Zhejiang University School of Medicine, Hangzhou, 310009 Zhejiang, China; ^2^Orthopedics Research Institute of Zhejiang University, Hangzhou, 310009 Zhejiang, China; ^3^Department of Breast Surgery, The Second Affiliated Hospital, Zhejiang University School of Medicine, Hangzhou, 310009 Zhejiang, China; ^4^Cancer Institute (Key Laboratory of Cancer Prevention and Intervention, China National Ministry of Education, Key Laboratory of Molecular Biology in Medical Sciences, Zhejiang Province), The Second Affiliated Hospital, Zhejiang University School of Medicine, Hangzhou, 310009 Zhejiang, China

## Abstract

**Background:**

This study is aimed at identifying the important biomarkers associated with bone metastasis (BM) in breast cancer (BRCA).

**Methods:**

The GSE175692 dataset was used to detect significant differential expressed genes (DEGs) between BRCA samples with or without BM, and DEG-related pathways were then explored. Further, we constructed the protein-protein interaction (PPI) network on GEGs and filtered 5 vital nodes. We then performed the Cox regression, Kaplan-Meier analysis, nomogram, and ROC curve to filter the most significant prognosis genes. The GSE14020 and GSE124647 datasets were used to verify the expression and prognostic value of hub genes, respectively. Finally, the gene set enrichment analysis (GSEA) was performed to reveal the potential mechanism.

**Results:**

Totally, 74 DEGs were detected, which mainly correlated with infectious disease, signaling molecules, and interaction. The 5 important DEGs were then filtered, and the Cox regression further showed that 2 genes, including prominin 1 (PROM1) and C-C motif chemokine ligand 2 (CCL2), were related to the prognosis of BRCA metastasis patients. Especially, PROM1 presented a better prognostic performance on the survival probability of patients than CCL2. Verification analysis further confirmed the abnormal expression and significant prognostic influence of PROM1. Finally, GSEA revealed that PROM1 was negatively related to IGF1 and mTOR pathways in BRCA metastasis.

**Conclusion:**

PROM1 was an important biomarker associated with BRCA bone metastasis and affected the prognosis of metastatic BRCA patients. It may play a vital role in metastatic BRCA by negatively regulating IGF1 and mTOR pathways.

## 1. Introduction

Metastasis accounted for more than 90% of cancer-related mortality [1]. The bone is one of the most preferred sites of metastatic spread from different cancer types, including breast cancer (BRCA). BRCA has become a critical health care issue that substantially affected women worldwide. Besides the lung, liver, and brain, the most common site for metastasis in BRCA is the bone [2]. The bone is also the first site of distant metastasis in 25% to 40% of patients with advanced BRCA [3]. It should be noted that different subtypes of BRCA exhibited distinct metastatic behavior in terms of kinetics and anatomic sites of relapse [4, 5]. For example, bone-only metastases were more common in the hormone receptor- (HR-) positive group than in the other subtypes [6]. The bone metastasis in BRCA was able to influence the survival of patients. It was reported that a 5-year survival rate of BRCA patients without metastasis was greater than 95% but close to only 20% once bone metastasis occurred [7]. In addition, BRCA bone metastasis also caused a series of bone-related complications such as pain, pathologic fractures, and spinal cord compression, which significantly affected the patient's quality of life [6], also increased the medical costs and mortality risk. As such, new targets and therapeutic strategies associated with BRCA bone metastasis are urgently required.

Over the past few decades, a great deal of biomarkers about BRCA bone metastasis has been generated, which facilitated the studies on cancer pathogenesis. Pantano et al. found that integrin alpha 5 (ITGA5) was highly expressed in bone metastases, compared to lung, liver, or brain metastases [8]. Awolaran et al. identified 15 proteins expressed by BRCA cells as factors that mediated BRCA bone metastasis, and upregulation of them could promote BRCA metastasis to bone, except for the C-C motif chemokine ligand 2 (CCL2) which showed a reduced expression [7]. Westbrook et al. identified and validated the dedicator of cytokinesis protein 4 (DOCK4) as a potential biomarker for risk of bone metastasis development in patients with early BRCA [9]. In addition, Zhang et al. found that microRNA-429 can inhibit BRCA bone metastasis by regulating matrix metallopeptidase 9 (MMP-9) [10]. More and more useful biomarkers should be detected to reveal the cancer pathogenesis involved in BRCA bone metastasis.

The present study was conducted to detect significant bone metastasis-associated biomarkers involved in BRCA. The differential expressed genes (DEGs) between BRCA bone metastasis and nonmetastatic samples were initially screened out through the Gene Expression Omnibus (GEO) dataset. Then, the impacts of significant DEGs on the survival probability of metastasis BRCA samples were predicted. Regarding significant prognostic biomarkers, we explored associated regulatory pathways involved in BRCA metastasis. This study was conducive to reveal useful biomarkers and potential mechanisms involved in BRCA bone metastasis.

## 2. Methods

### 2.1. DEG Identification and Function Analysis

The proper dataset for screening the differential expressed genes (DEGs) was selected from the Gene Expression Omnibus (GEO) database (https://www.ncbi.nlm.nih.gov/geo/). Finally, the GSE175692 dataset which contained 33 BRCA bone metastasis samples and 151 nonbone metastasis samples was used to detect significant DEGs. According to the threshold of *P* < 0.05 and absolute log fold change (FC) > 1, the DEGs between the 2 groups were identified by the limma R package. And the top 20 up- and downregulated DEGs were presented. Subsequently, the significant Kyoto Encyclopedia of Genes and Genomes (KEGG) pathway and Gene Ontology (GO) terms about DEGs were explored through the clusterProfiler R package. GO terms were annotated from the biological process (BP), cellular component (CC), and molecular function (MF) aspects.

### 2.2. PPI Network Construction and Hub Genes Determination

The protein-protein interaction (PPI) network among DEGs was constructed using the online tool String (https://cn.string-db.org/) setting the interacting score as medium, followed by visualization through Cytoscape. The top 10 hub genes among the whole PPI network were detected by the degree gene ranking method using the Cytohubba plug-in of Cytoscape. The Venn analysis was then performed to filter overlapped nodes between the top 10 hub genes and top 20 DEGs. Finally, 5 consistent nodes were identified for further investigation.

### 2.3. Expression and Prognosis Analysis on Hub Genes

Differential expression of 5 hub genes between BRCA samples with or without bone metastasis was firstly evaluated using the dataset of GSE175692. Prognosis associated hub genes in BRCA metastasis was then evaluated through the univariate Cox regression analysis. The Kaplan-Meier analysis was performed to explore the influence of hub genes expression on the overall survival of BRCA metastasis samples. Further, nomogram and receiver operating characteristic (ROC) curve analyses were conducted to reveal the prognostic performance of hub genes. Through a series of filtration, the 2 most important hub genes (C-C motif chemokine ligand 2 (CCL2) and prominin 1 (PROM1)) were finally identified.

### 2.4. Expression and Prognostic Value Verification on Hub Genes

Regarding the most important hub genes, the GSE14020 dataset which contained 18 bone metastasis and 47 nonbone metastasis BRCA samples was used to verify their mRNA expression. Moreover, the prognostic value of 2 hub genes on the overall survival of BRCA metastasis patients was also verified by the Kaplan-Meier analysis using the GSE124647 dataset which included 140 BRCA metastasis samples.

### 2.5. GSEA on Significant Prognostic Factors

Due to the differential expression and vital prognostic effect of significant prognostic factors in metastasis BRCA samples, we performed the gene set enrichment analysis (GSEA) to explore the possible mechanism associated with BRCA metastasis. The gene expression profile for GSEA was obtained from the GSE175692 dataset which included 184 BRCA metastasis samples. All the patients were divided into high and low expression groups according to the median gene expression level. Then, the potential pathway enriched in high-/low-expression groups was predicted by GSEA. The threshold for GSEA was set as follows: the number of permutations (1000), enrichment statistic (weighted), and metric for ranking genes (Pearson).

### 2.6. Statistical Analysis

The expression difference between the 2 groups was compared with the independent-samples *t*-test or Mann–Whitney test, and the results were presented with the violin chart and box scatter which contained the expression median, upper quartile, lower quartile, maximum, and minimum. The effects of gene expression on the survival of patients were evaluated through survival analysis and Cox regression showing hazard ratio (HR) and 95% confidence interval (CI). *P* < 0.05 was considered statistical significance.

## 3. Results

### 3.1. DEGs Identification and Function Analysis

The GSE175692 dataset was used to filter the DEGs between BRCA samples with or without bone metastasis. A total of 74 significant DEGs were found according to absolute LogFC > 1 and *P* value < 0.05, and the top 10 upregulated and 10 downregulated DEGs were marked (Figure 1(a)). The KEGG analysis showed that 74 DEGs were mainly associated with infectious disease, signaling molecules, and interaction (Figure 1(b)). The enriched pathway of partial DEGs is shown in Figure 1(c).

Functional enrichment analysis was then performed to reveal the role of 74 DEGs in cancer progression (Figure 2). The significant enriched KEGG pathway included ECM-receptor interaction, cytokine-cytokine receptor interaction, and human papillomavirus infection. For cellular component, the DEGs were largely located at the collagen-containing extracellular matrix and extracellular matrix. For biological process, DEGs primarily participated in extracellular structure organization. In terms of molecular function, DEGs were significantly enriched in receptor regulator activity and receptor ligand activity.

### 3.2. Hub Gene Determination and Differential Expression Analysis

The protein-protein interaction (PPI) network among DEGs was constructed using String and Cytoscape. The PPI network contained 60 nodes and 167 edges (Figure 3). Using the degree gene ranking method, we identified the top 10 hug genes, namely the estrogen receptor 1 (ESR1), matrix metallopeptidase 9 (MMP9), bone morphogenetic protein 2 (BMP2), secreted phosphoprotein 1 (SPP1), C-C motif chemokine ligand 2 (CCL2), progesterone receptor (PGR), Wnt family member 2 (WNT2), matrix metallopeptidase 3 (MMP3), integrin subunit beta 3 (ITGB3), and prominin 1 (PROM1).

The consistent genes between the top 20 DEGs and 10 hub genes were determined. The 5 most significant hub genes were subsequently found, which contained 3 upregulated (MMP9, ITGB3, and BMP2) and 2 downregulated (CCL2 and PROM1) DEGs (Figure 4(a)). The detailed information of 5 hub genes in GSE175692 is presented in Figure 4(b). Differential expression of 5 hub genes between bone metastasis and nonbone metastasis BRCA samples was then compared (Figure 4(c)), and results showed that 5 hub genes were abnormally expressed in BRCA bone metastasis group compared with that in the nonbone metastasis group.

### 3.3. Prognostic Value Analysis on Hub Genes

We firstly performed the univariate Cox regression to screen the prognosis-related biomarkers in metastatic BRCA and found that PROM1 and CCL2 showed a significant correlation with the overall survival of patients (Figure 5(a)). Survival analysis indicated that high expression of PROM1 and CCL2 shortened the overall survival time of metastatic BRCA patients (Figure 5(b)). We also explored their prognostic impacts on the survival of BRCA patients with single bone metastasis. However, both PROM1 and CCL2 exerted no significant impacts on the survival of single BRCA bone metastasis patients (Figure 5(c)), which might be due to the insufficient sample size.

Subsequently, the prognostic performance of PROM1 and CCL2 in metastatic BRCA was evaluated. A nomogram analysis showed that PROM1 possessed the largest contribution to the survival probability of patients, contributing 100 points (Figure 6(a)). The ROC analysis indicated that the prediction ability of PROM1 was slightly superior to CCL2 (Figure 6(b)).

### 3.4. Expression and Prognostic Value Verification of Hub Genes

The above results indicated the significance of PROM1 and CCL2 in metastatic BRCA; we further verified their expression and prognostic value in metastatic BRCA. Quantitative analysis just revealed the significant expression difference of PROM1 between BRCA samples with or without bone metastasis (Figure 7(a)). The survival analysis (Figure 7(b)) also showed the significant prognostic impact of PROM1 on the patients. Verification analysis further disclosed the significance of PROM1 in metastatic BRCA.

### 3.5. GSEA on PROM1

PROM1 was determined as a vital downregulated gene in bone metastasis and played an important role in metastasis BRCA progression. Finally, we explored the potential mechanism of PROM1 involved in metastasis BRCA. The GSEA indicated that PROM1 was negatively associated with insulin-like growth factor 1 (IGF1) and mechanistic target of rapamycin kinase (mTOR) pathways (Figure 8). We speculated that PROM1 might influence metastasis BRCA development through negatively regulating IGF1 and mTOR pathways.

## 4. Discussion

It has been reported that 70% of patients with metastatic BRCA have a marked tendency to spread to the bone, resulting in significant skeletal complications and mortality [11]. Despite advances in diagnosis, the identification of patients at high risk of bone recurrence is still an unmet clinical need. Therefore, identifying useful biomarkers was conducive to improve the clinical outcome of metastatic BRCA patients. Spadazzi et al. have identified trefoil factor 1 (TFF1) as strictly correlated to bone metastasis from estrogen receptor (ER) + breast cancer, and TFF1 upregulation could be useful to identify patients at high risk of bone metastasis [12]. Pantano et al. determined integrin subunit alpha 5 (ITGA5) as a predictive of poor bone metastasis-free survival [8]. As the bone is the most frequent organ for breast cancer metastasis, thus it is essential to predict the bone metastasis of breast cancer.

In this study, we firstly identified 74 significant DEGs between BRCA samples with or without bone metastasis. These 74 DEGs mainly participated in ECM-receptor interaction and cytokine-cytokine receptor interaction, which referred to signaling molecules and interaction. The previous study has indicated that ECM-receptor interaction significantly participated in breast cancer metastasis to the bone [13] and brain [14]. The ECM-receptor interaction pathway was also correlated to lung metastasis in osteosarcomas [15], lung adenocarcinoma metastasis [16], and liver metastasis of colorectal cancer [17]. In addition, virus infection such as human papillomavirus (HPV) infection was also proved to correlate with DEGs in our study. During the last decades, great interest has been given to the viral pathogenesis of breast cancer. Habyarimana et al. showed that human papillomavirus (HPV) DNA was found in 46.81% of Rwandese breast cancer cases, HPV16 being the most prevalent subtype (77.27%) followed by HPV33 (13.64%) and HPV31 (9.09%) [18], suggesting high-risk HPV infections as a risk factor in breast cancer development. Cavalcante et al. found that the high frequency of HPV infection in breast cancer samples indicated a potential role in breast carcinogenesis [19]. However, Hedau et al. found no evidence of HPV pathogenesis of breast cancer in Indian women [20]. And the low frequency of HPV was detected in Ghaffari et al.'s study, which also did not support the association between breast carcinoma and HPV infection [21]. It followed that effect of HPV infection in BRCA was not uniform, and it was possible that HPV may be responsible for breast carcinogenesis only in a small percentage of all breast cancer.

Subsequently, we found the 5 most important hub genes among all GEGs, namely MMP9, ITGB3, BMP2, CCL2, and PROM1. A univariate Cox regression initially identified that PROM1 and CCL2 expressions were related to the prognosis of metastatic BRCA patients. Survival analysis, nomogram, and ROC curve analyses further presented the significance of PROM1 on the survival probability in metastatic BRCA. Expression analysis showed that PROM1 was upregulated in BRCA bone metastasis samples compared with no bone metastasis samples. The above results showed that PROM1 was an important DEGs involved in bone metastasis of BRCA and presented a good prediction performance on the patient's survival probability.

Prominin 1 (PROM1), also called CD133, is a transmembrane glycoprotein which is expressed in stem cell lineages [22]. The importance of PROM1 in BRCA has been reported. Priedigkeit et al. reported that PROM1 was related to transcriptional remodeling in long-term estrogen-deprived locoregional breast cancer recurrences [23]. Bertheau et al. identified PROM1 as a mutant TP53-associated gene involved in breast cancer [24]. Xia analyzed the prognostic roles of PROM1 mRNA in the subtypes of BRCA and concluded that PROM1 mRNA may be a suitable prognostic marker for human BRCA [25]. Liu et al. found that PROM1 was not expressed in the cells of normal breast tissue, but the expression rate increased with progression of lesions from usual hyperplasia, through atypical ductal hyperplasia, ductal carcinoma in situ, and invasive carcinoma, suggesting that PROM1 positive breast cancer cells were closely related to invasiveness and its expression may predict a poor prognosis [26]. Bock et.al found that N-cadherin and PROM1 expressions were strongly correlated, which suggested the role of PROM1 in the migration of breast cancer [27]. Regarding the bone metastasis of BRCA, Leni et al. indicated that PROM1 showed a highly significant value regarding metastatic localizations in the bone [28]. At present, few studies reported the role of PROM1 in the BRCA bone metastasis, and more investigations are needed to be performed in the future.

This study has indicated the important function of PROM1 in BRCA metastasis, and we finally explored the potential mechanism associated with PROM1. GSEA indicated that PROM1 was significantly related to mTOR and IGF1 pathways with a negative correlation. The mTOR critically regulated several essential biological functions, such as cell growth, metabolism, survival, and immune response [29]. However, the mTOR was frequently deregulated in human cancers [30]. It has demonstrated that PROM1 played a key role in the regulation of autophagy via upstream suppression of mTOR signaling in the human retinal pigment epithelium [22]. Kholodenko et al. found that cells with the complete knockout of PROM1 showed the highest resistance to mTOR inhibitors in colorectal cancer [31]. Our study suggested that low expression of PROM1 might activate the mTOR pathway in BRCA metastasis samples.

IGF are the most abundant growth factors in bone and are required for normal skeletal development and function. Via activation of the IGF1 receptors (IGF1R) and variant insulin receptors, IGFs promote cancer progression, aggressiveness, and treatment resistance [32]. Preclinical evidence has suggested that a high IGF1 environment in primary tumor stimulated tumor cells metastasis to bone, suggesting that bone metastases may reflect IGF dependency [32]. Several studies have indicated that IGF signaling systems were able to regulate BRCA growth, progression, and metastasis [33, 34]. It followed that the IGF1 pathway played a vital function in the progression of BRCA metastasis. However, this study just indicated the negative correlation between PROM1 and IGF1/mTOR pathways; the detailed regulation in BRCA metastasis especially bone metastasis was worth further investigating.

There are limitations that consist in this article. First, PROM1 expression in clinical samples should be detected by qPCR or IHC, and its prognostic significance needs to be further confirmed in clinical cases. Second, we have explored the potential pathways associated with PROM1 with the public databases, but how PROM1 modulates mTOR and IGF1 pathways in metastasis BRCA remains unclear, and both in vivo and in vitro experiments need to be investigated.

## 5. Conclusion

This study identified 74 DEGs between BRCA samples with or without bone metastasis, and 5 important DEGs were finally filtered, namely, MMP9, ITGB3, BMP2, CCL2, and PROM1. Through the Cox regression and Kaplan-Meier survival analysis, PROM1 and CCL2 were determined as the significant prognosis-related biomarkers associated with metastatic BRCA. Prognosis verification analysis further indicated the importance of PROM1 rather than CCL2. Especially, both nomogram and ROC analyses presented the better prediction ability of PROM1 on the survival probability of metastatic BRCA patients. Finally, we found that PROM1 negatively correlated with IGF1 and mTOR pathways involved in BRCA metastasis. This study identified PROM1 as an important prognosis-related biomarker associated with metastatic BRCA, and detailed function needed further investigation via experimental verification and clinical cohort.

## Figures and Tables

**Figure 1:** The DEG identification and mechanism exploration. (a) Volcano plot and top 20 DEGs presentation. (b) KEGG pathway and classification. (c) Correlation between the DEG and KEGG pathway. Abbreviation: DEGs: differential expressed genes; KEGG: Kyoto Encyclopedia of Genes and Genomes.

**Figure 2:** Functional enrichment analysis on 74 DEGs containing the KEGG pathway and GO annotation. Abbreviation: DEGs: differential expressed genes; KEGG: Kyoto Encyclopedia of Genes and Genomes; GO: Gene Ontology.

**Figure 3:** The PPI network among DEGs. Green nodes indicated the top 10 hub genes identified by the degree method. Abbreviation: DEGs: differential expressed genes; PPI: protein-protein interaction network.

**Figure 4:** Significant hub genes determination and expression analysis. (a) The Venn analysis for determining more important hub genes. (b) Detailed information of 5 hub genes in GSE175692. (c) The mRNA expression of 5 hub genes in BRCA samples with or without bone metastasis in the GSE175692 dataset. Abbreviation: BRCA: breast cancer.

**Figure 5:** The prognostic value analysis of hub genes on the overall survival of metastatic BRCA samples in GSE175692. (a) Cox regression for predicting prognostic factors associated with BRCA metastasis. The effects of gene expression on the overall survival of (b) metastatic samples and (c) single bone metastasis samples. Abbreviation: BRCA: breast cancer.

**Figure 6:** Prognostic performance analysis on PROM1 and CCL2 in metastatic BRCA in GSE175692. (a) Nomogram. (b) ROC curve. Abbreviation: BRCA: breast cancer; ROC: receiver operating characteristic; AUC: area under curve; CCL2: C-C motif chemokine ligand 2; PROM1: prominin 1.

**Figure 7:** The expression and prognostic value verification of PROM1 and CCL2. (a) Differential expression of hub genes between BRCA bone metastasis and nonbone metastasis samples (GSE14020). (b) The Kaplan-Meier survival analysis (GSE124647). Abbreviation: BRCA: breast cancer; CCL2: C-C motif chemokine ligand 2; PROM1: prominin 1.

**Figure 8:** GSEA on PROM1 in metastasis BRCA samples using the GSE175692 dataset. Abbreviation: BRCA: breast cancer; GSEA: gene set enrichment analysis; PROM1: prominin 1.

## Data Availability

The datasets used and/or analyzed during the current study are available from the corresponding author on reasonable request.
